# Multipath Cross Graph Convolution for Knowledge Representation Learning

**DOI:** 10.1155/2021/2547905

**Published:** 2021-12-28

**Authors:** Luogeng Tian, Bailong Yang, Xinli Yin, Kai Kang, Jing Wu

**Affiliations:** ^1^High-Tech Institute of Xi'an, Xi'an 710025, China; ^2^Information and Communication College, National University of Defense Technology, Xi'an, 710106, China; ^3^National Innovation Institute of Defense Technology, Beijing 100071, China

## Abstract

In the past, most of the entity prediction methods based on embedding lacked the training of local core relationships, resulting in a deficiency in the end-to-end training. Aiming at this problem, we propose an end-to-end knowledge graph embedding representation method. It involves local graph convolution and global cross learning in this paper, which is called the TransC graph convolutional network (TransC-GCN). Firstly, multiple local semantic spaces are divided according to the largest neighbor. Secondly, a translation model is used to map the local entities and relationships into a cross vector, which serves as the input of GCN. Thirdly, through training and learning of local semantic relations, the best entities and strongest relations are found. The optimal entity relation combination ranking is obtained by evaluating the posterior loss function based on the mutual information entropy. Experiments show that this paper can obtain local entity feature information more accurately through the convolution operation of the lightweight convolutional neural network. Also, the maximum pooling operation helps to grasp the strong signal on the local feature, thereby avoiding the globally redundant feature. Compared with the mainstream triad prediction baseline model, the proposed algorithm can effectively reduce the computational complexity while achieving strong robustness. It also increases the inference accuracy of entities and relations by 8.1% and 4.4%, respectively. In short, this new method can not only effectively extract the local nodes and relationship features of the knowledge graph but also satisfy the requirements of multilayer penetration and relationship derivation of a knowledge graph.

## 1. Introduction

With the increasing construction of giant knowledge graphs, graph neural networks (GNNs), graph convolutional network (GCN) [1], and other neural networks that originally performed well on the graph appear to be incapable, and the calculation of adjacency matrix with full graph has become a problem. In many task scenarios, the entities in the map have close and important relationships with surrounding entities [2–4] and may have nothing to do with entities beyond a few steps. For example, TransE [5] series mostly only consider the direct relationship between entities. However, facts show that the rich and complex multistep relationships between entities in the knowledge graph are of great value for improving the quality of knowledge graph embedding. In a sense, the value of an entity lies in its interaction with other entities. This relationship can be quantitative or qualitative. In other words, the same entity has relatively stable characteristic attributes in a fixed scene, and the relationship path is the necessary information supplement of the entity. The multilayer type of the entity mapped by its relationship is significant in knowledge representation learning or logical reasoning [6]. Moreover, various works have also been developed that support entity and relationship prediction [7–9]. For example, Hogan [10] replaced entities with canonical labels for solemnising existential nodes. Zhao et al. [11] proposed an effective method of using local relationships in entity type prediction.

A large number of knowledge graph cases show that a node often has a strong semantic relationship with a small number of adjacent nodes. It is not like GCN on “seeing flowers in the fog” and “finding needles in the sea” on the entire map, learning some valuable information from the giant knowledge map. Through the training and learning of the model, we should enable it to accurately classify the types of entities and predict and judge the attributes of the classified entities. An example is shown in Figure 1<LeBron Raymone James, player number, ？>.

The simple dot product of feature vectors and linear classification calculations can cause certain feature loss, which makes the entity classification and attribute prediction ineffective. As such, we propose a lightweight GCN for nonlinear cross learning of local knowledge graphs. Global iteration will certainly improve the coverage and accuracy, but this is often at the expense of the computational efficiency of the algorithm. At the same time, the knowledge graph structure or the baseline models of knowledge representations, such as TransE, TransR [12], and PTransE [13], considers the 1–3 step relationships and proves that the algorithm's reasoning performance can be improved [14].

Given an example of such a set of triples as in Figure 2:<Titanic, leading actress, Kate Winslet>< Avatar, leading actress, Zoe Saldana>< Zoe Saldana, bra, Athletic undergarment><James Cameron, cooperative partner, LeBron Raymone James>< LeBron Raymone James, play for, Los Angeles Lakers>< LeBron Raymone James, another name, LBJ><LeBron Raymone James, another name, Zhan Huang><LeBron Raymone James, wife, Savannah James><LeBron Raymone James, player number, 23>.

To sum up, PTransE has a significant impact on the relational path embedding. It integrates multistep relational paths into knowledge representation learning, realizes information reasoning from the relational level, and improves the performance of knowledge graph completion. In terms of path selection, we proposed a resource allocation algorithm. Although this algorithm is feasible in quickly obtaining an effective relationship path, it is easy to cause resources to move closer to the entity that flows to the first step. If we select the first step of resource flow to the entity path, the first step of relationship path fitting will be generated. The main reason is that the co-occurrence relationship of global node features is ignored. Thus, a new local convolution global crossover named TransC-GCN is proposed in this study. It can not only effectively extract the local nodes and relationship features of the knowledge graph but also consider the needs of multilayer penetration and relationship derivation of the knowledge graph.

We are committed to embedding giant graphs and high-dimensional entities into low-dimensional entity type relationships.  Figure 3 presents an example of learning and crossing through multiple local semantic spaces with similar classes, finally achieving two goals: (1) entity type judgment and classification and (2) entity name prediction.

Based on the research goals, we consider further adding local knowledge relationship path features on the basis of PTransE. At the same time, we combine multiple local crosses to realize the combination of local deep learning of relationship paths and global fusion representation.

  Through the graph convolution learning of local entity relationship, not only can the hidden entities and relationship features in the local be discovered but also the local knowledge representation effect can be improved.
  The continuous improvement of local knowledge representation ability will improve the overall knowledge learning performance and strengthen the knowledge reasoning ability.
  The small-scale local graph convolution application can avoid the occurrence of global overfitting while solving the long calculation time.

In order to achieve the above goals, we need to address two challenges:

1. *Partial Division Problem*. If the part is too small, it will increase the amount of graph convolution calculation. On the contrary, the local features would be too rough. Therefore, partial division is the primary challenge.
2. *Cross Loss Function*. The iterative application of the local GCN improves the learning effect of local features by defining the loss function and constraining the optimization during the local crossover process. This is a key to ensuring the quality of the model.

Our contributions can be summarized as follows:

1. Using graph convolution combined with the out degree and in degree of the knowledge graph to iteratively calculate the local range, which can prevent the local division from being too large, we limit the local calculation to a certain threshold range related to the global graph structure.
2. The joint loss function is constructed through knowledge prior probability, posterior probability, and local cross entropy, which is calculated by normalization.

## 2. Related Works

### 2.1. GCN Full Graph Reasoning

Kipf et al. [15] introduced Spectral GCNs for semisupervised classification of spatial GCN graph structure data and applied convolution operations to calculate new feature vectors for each node with its neighborhood information. The fly in the ointment is that GCN needs to import the entire image to train the information and requires the training data to be unified with the verification data.

GCN combining features of nearby nodes is dependent on the structure of the graph, which limits the generalization ability of the trained model on other graph structures. Ermis et al. [16] believe that in a graph, predicting the link relationship between nodes can better study the entire graph network. For example, Wu et al. [17] used GCN to express the relationship between users and projects in the user-project structure diagram. Wang et al. [18] used GCN in KGs to improve the recommendation effect, while causing the hidden danger of overfitting and GCN performance degradation due to the lack of regularization. Wang et al. [19] realized the alignment of cross language knowledge graphs through graph convolutional networks.

### 2.2. Neighbor Sampling Learning

Graph Sample and Aggregate (GraphSAGE) is the most representative method in terms of uniform sampling of neighbor nodes and local node aggregation, as shown in Figure 4. By training the function of neighbors on the aggregated subgraph nodes, GCN is extended to inductive learning, thereby generalizing unknown nodes [18].

GAT [20] uses the attention distribution metric of neighbor nodes to weight and aggregate the local implicit information of the adjacency matrix. The local graph embedding representation of the central node is composed of the feature representation of the central node and that of neighbor nodes. Through the splicing of node vectors, the feature representation of the center node can be iteratively updated, and then the feature representation of all nodes on the graph can be updated. In essence, GAT uses the feature aggregation function of the attention weight of neighbor nodes instead of the normalized function of GCN.

Unlike GCN, GAT allows implicitly assigning different importance to neighbors of the same node, while learning that attention is helpful for the interpretability of the model. The operation of GAT is point-by-point, and it is unnecessary to visit the global graph structure in advance. Therefore, it is suitable for inductive tasks. Important nodes in the graph and relations between nodes help to filter the noise between the neighbors of nodes and improve the interpretability of model results.

### 2.3. Embedding

A wide range of knowledge graph embedding techniques has been proposed. Based on the idea of TransE, the Trans(D,R) [21] defines the projection matrix *M*_*r*_ for the relationship *r* of each triplet *<h*, *r*, *t>* from the perspective of the relationship difference, and the head and tail entities are projected into the corresponding relational space. Then, TransE is used for translation. It is just that the head entity and the tail entity share *M*_*r*_ in the same triple, and there is no distinction between the head entity and the tail entity.

For example, <LeBron Raymone James, work for, Los Angeles Lakers>, LeBron Raymone James is a person's name, and Los Angeles Lakers represents the collective. According to the above methods, we find that < James Cameron, director, Titanic> and <James Cameron, director, Avatar > are two triples with the same head entity and relationship. So, their tail entities are Titanic ≈ Avatar. Obviously, this is incompatible with the fact. To solve this problem, TransD considers the difference between the head and tail entities. Similar to TransR, the head and tail entities are respectively projected into the relation *r* space; then, *M*_*rh*_*h* and *M*_*rt*_ are obtained. CrossE [22] uses a relational interaction matrix *C* to generate the interaction vector of the head entity and the relationship and then uses the vectors of these two interaction representations to predict the tail entity.

## 3. Algorithm Model

In this section, we propose an end-to-end knowledge map convolutional cross embedding representation method (TransC-GCN) as shown in Figure 5. Firstly, multiple local semantic spaces are divided according to the largest neighbor, and then a translation model is used to map the local entities and relationships into a cross vector, which is used as the input of GCN. Through training and learning of local semantic relations, the best entity and the strongest relationship are found. Finally, the optimal entity relationship combination output is evaluated through the posterior loss function based on the mutual information entropy.

The framework is mainly composed of 4 parts: (1) partial knowledge graph learning partitioning and embedding representation; (2) performing GCN coding on the partial graph and using the combined node relationship of the partial graph as input; (3) cross aggregating multiple partial knowledge graphs along with key relationships into reasoning nodes; and (4) sorting prediction nodes for multiple relationship paths.

### 3.1. Subgraph Division

There are often complex relationships between nodes in a local knowledge graph. Therefore, the minibatch method is used for reference to the set of local subgraphs, which is composed of central nodes. Besides, all nodes at the *q*-order subgraph of ℬ are presampled and stored in the traversal. Feature and label propagation are only propagated in the local map. So, we define the subgraph division as follows.

**Definition 1 .**

Given *G*={*E*, *R*}, assume |*ℰ*|=*n*, |ℛ|=*m*. Define its incidence matrix  A ∈ ℝ^*n*×*m*^ as follows:

(1) $$\begin{array}{c} r_{ij}=\left\{\begin{array}{cc} 1, & i\in E_{j},\\ 0, & i\notin E_{j}. \end{array}\right. \end{array}$$

**Definition 2 .**

The number of nodes is *n* < *∞*. Use one  *n* × *n*  matrix to represent adjacency matrix *G*, which is defined as *A*(*G*)=(*a*_*i*,*j*_), where *n* is the order of the graph. The set of **A**(*G*) features is called spectrum of the graph.

(2) $$\begin{array}{c} a_{i,j}=\left\{\begin{array}{cc} 1, & \left(i,j\right)\in E,\\ 0, & \text{other}. \end{array}\right. \end{array}$$

**Definition 3 .**

 *G*_*c*_={*E*_*c*_, *R*_*c*_}  represents a subgraph of the knowledge graph used for cross learning *c*, where *E*_*c*_ is a collection of head and tail entities in the subgraph of *C* and **ℛ**_*c*_ is the collection of relations among all nodes. Neighbor nodes of *e*_*i*_^(*c*)^ are defined as N(*e*_*ij*_^(*c*)^)={*D*(**e**_*i*_^(*c*)^, **e**_*j*_^(*c*)^) ≥ *d*°}.

(3) $$\begin{array}{c} D\left(e_{i}^{\left(c\right)},e_{j}^{\left(c\right)}\right)=\frac{1}{1+\left\|e_{i}^{\left(c\right)}-e_{j}^{\left(c\right)}\right\|}, \end{array}$$

(4) $$\begin{array}{c} d^{\circ }=\frac{1}{\left|C\right|}\overset{\left|C\right|}{\underset{j=1}{\sum }}{\left\|e_{i}^{\left(c\right)}+r^{\circ }-e_{j}^{\left(c\right)}\right\|}_{\ell 2}^{2}, \end{array}$$

where *D*(**e**_*i*_^(*c*)^, **e**_*j*_^(*c*)^) denotes the Euclidean distance between the center node *i* to the neighbor node *j* and *d*° is the relational path threshold of global graph. A local subgraph about the central node *i* is defined as *𝒮*_*i*_^(*c*)^. The schematic diagram of process is shown in Figure 6.  Algorithm 1 shows the details of the calculation process.

### 3.2. Local Relation Graph Convolutional Coding

GCN can obtain the local information more accurately. Maximum pooling operation helps to grasp the strong signal on the local feature, thereby avoiding noise interference of the global redundant feature. Average pooling is used for neurons. The neighbor nodes connected to the central node are embedded as the input of a layer of neural network. Average pooling is used to eliminate the sparseness or overfitting problems of local nodes and relationship features. So, we use a layer of fully connected neural network and maximum pooling. Then, the output vector is multiplied by the feature vector of the central node to obtain a local embedding representation.

(5) $$\begin{array}{c} Y_{out}\left(G_{c}\right)=\overset{M}{\underset{m=1}{\sum }}D_{m}^{-1/2}{\hat{A}}_{m}D_{m}^{-1/2}XW_{m}^{\left(\ell \right)}, \end{array}$$

(6) $$\begin{array}{c} {\hat{A}}_{m}=A_{m}+I_{m}. \end{array}$$

The connection matrix ${\hat{A}}_{m}$ is the label of *m*, *m* ∈ {1,2,…, *M*}, and **D**_*m*_^−1/2^ is the degree matrix corresponding to ${\hat{A}}_{m}$.

(7) $$\begin{array}{c} \alpha_{ij}^{\left(c\right)}=\frac{exp\left(\text{LeakReLU}\left(\left(W_{h}^{\left(\ell \right)}H_{c}^{\left(\ell \right)}+b_{s}\right)+\epsilon^{{}^{\circ}}\right)\right)}{\sum_{k\in }exp\left(\text{LeakReLU}\left(\left(W_{h}^{\left(\ell \right)}H_{c}^{\left(\ell \right)}+b_{s}\right)+\epsilon^{{}^{\circ}}\right)\right)}, \end{array}$$

where *α*_*ij*_^(*c*)^=(*α*_*i*1_^(*c*)^, *α*_*i*2_^(*c*)^, ⋯, *α*_*ic*_^(*c*)^),  **W**_*h*_^(*ℓ*)^ is the weight matrix between hidden layers, and  *b*_*s*_ and *ϵ*° are the deviations. The nonlinear activation function *σ* is *ReLU*.  Figure 7 shows the partial relationship diagram of the convolutional coding process.

### 3.3. Graph Relational Cross Matrix

In order to eliminate the overfitting of some important relationship nodes caused by the division of local graphs, multiple heads can be used to calculate *C* subgraph branches in parallel. Then, all the subgraph branches can be defined by

(8) $$\begin{array}{c} {\bar{\alpha }}_{ij}^{c}=\frac{1}{\left|C\right|}\underset{j\epsilon N_{i}}{\sum }\alpha_{ij}^{C}. \end{array}$$

Local cross matrix:

(9) $$\begin{array}{c} C_{\alpha }=C_{\alpha }C_{\alpha }^{T}=\left[{\bar{\alpha }}_{ij}^{1},{\bar{\alpha }}_{ij}^{2},\ldots ,{\bar{\alpha }}_{ij}^{m}\right]{\left[{\bar{\alpha }}_{ij}^{1},{\bar{\alpha }}_{ij}^{2},\ldots ,{\bar{\alpha }}_{ij}^{m}\right]}^{T}=\left[\begin{array}{ccc} c_{11} & \cdots & c_{1m}\\ \vdots & \ddots & \vdots \\ c_{m1} & \cdots & c_{mm} \end{array}\right]. \end{array}$$

**Definition 4 .**

The graph cross matrix scaling factor is defined by the matrix mutual interference parameter [23], which measures the mutual interference parameters between different column vectors of local cross matrix. Specifically, the similarity relationship between the local graph structures can be found:

(10) $$\begin{array}{c} \rho =\underset{i\neq j}{\max}\left|c_{i},c_{j}\right|=\underset{i\neq j}{\max}\left|c_{i}^{H},c_{j}\right|. \end{array}$$

From (9) and (10), the graph cross matrix of the fusion local graph structure is given by **C**=*ρ ***C**_*α*_.

### 3.4. Dynamic Node Prediction

The normalized attention coefficient is used to sum the weighted features as the preliminary output feature of each node:

(11) $$\begin{array}{c} {\overset{⟶}{e}}_{i}^{\prime }=ReLU\left(\underset{j\epsilon N_{i}}{\sum }\alpha_{ij}W{\overset{⟶}{e}}_{j}\right), \end{array}$$

(12) $$\begin{array}{c} {\overset{⟶}{e}}_{i}^{\prime }=ReLU\left(\frac{1}{\left|C\right|}\overset{\left|C\right|}{\underset{c=1}{\sum }}\underset{j\epsilon N_{i}}{\sum }{\bar{\alpha }}_{ij}^{c}W^{\left(\ell \right)}{\overset{⟶}{e}}_{j}\right). \end{array}$$

Local subgraph prediction node output:

(13) $$\begin{array}{c} {\hat{Y}}_{\mathrm{ci}}\left(e_{ij}^{\left(c\right)}\right)=\underset{ij\in N\left(e_{ij}^{\left(c\right)}\right)}{\sum }\frac{1}{S_{i}^{\left(c\right)}\left(e_{j}^{\left(c\right)}\right)}X\left(e_{j}^{\left(c\right)}\right)W^{\left(\ell \right)}\left(e_{j}^{\left(c\right)}\right), \end{array}$$

where **X**(*e*_*j*_^(*c*)^) is the characteristic of *e*_*j*_^(*c*)^;  **W**^(*ℓ*)^  is *e*_*j*_^(*c*)^  with GCN of shared weights on *ℓ*th layer; *𝒮*_*i*_^(*c*)^ is the normalized subset corresponding to all adjacent nodes *𝒩*(*e*_*j*_^(*c*)^) of *e*_*i*_^(*c*)^; and ${\hat{𝒴}}_{\mathrm{ci}}\left(e_{ij}^{\left(c\right)}\right)$ is the target representation vector centered on *e*_*i*_^(*c*)^.

### 3.5. Loss Function

#### 3.5.1. Triple Knowledge Embedding Loss Function

Cross correlation score of entities and relationships within triplet is used as the object of knowledge representation optimization. Here, the formal scoring function is given by

(14) $$\begin{array}{c} {ℒ}_{Emb}=-\underset{\left({\text{e}}_{i}^{\left(c\right)},r_{ij}^{{}^{\circ}},{\text{e}}_{j}^{\left(c\right)}\right)}{\sum }\left[\log\;Pr\left({\text{e}}_{i}^{\left(c\right)}|{\text{r}}_{ij}^{{}^{\circ}},{\text{e}}_{j}^{\left(c\right)}\right)+\text{log}Pr\left({\text{e}}_{j}^{\left(c\right)}|{\text{e}}_{i}^{\left(c\right)},{\text{r}}_{ij}^{{}^{\circ}}\right)+\log\;Pr\left({\text{r}}_{ij}^{{}^{\circ}}|{\text{e}}_{i}^{\left(c\right)},{\text{e}}_{j}^{\left(c\right)}\right)+\theta_{1}^{{}^{\circ}}\right]. \end{array}$$

#### 3.5.2. Cross Convolution Loss Function

A graph convolution operator is inside the local knowledge graph, and multiple local graphs are cross fused based on the information divergence. The local knowledge map features learned from the local convolution model are fed into the divergence fusion cross model. At the same time, we use gradient optimization algorithms of AdaGrad and stochastic gradient descent (SGD) to construct training modules. The estimated difference of partial subgraph output is defined as follows:

(15) $$\begin{array}{c} \underset{N}{\min}{ℒ}_{GCN}=C_{JS\;D}\left(Y_{ci},{\hat{Y}}_{\mathrm{ci}}\right)\\ =KL\left(Y_{ci}\frac{Y_{ci}+{\hat{Y}}_{\mathrm{ci}}}{2}\right)+KL\left({\hat{Y}}_{\mathrm{ci}}\frac{Y_{ci}+{\hat{Y}}_{\mathrm{ci}}}{2}\right)+\theta_{2}^{{}^{\circ}}\\ =\underset{i\in A}{\sum }Y_{ci}\left[\log\frac{Y_{ci}}{{\hat{Y}}_{\mathrm{ci}}}\right]+\underset{i\in B}{\sum }{\hat{Y}}_{\mathrm{ci}}\left[\log\frac{{\hat{Y}}_{\mathrm{ci}}}{Y_{ci}}\right]+\theta_{2}^{{}^{\circ}}. \end{array}$$

The loss function of global cross training error rate for the supervised training optimization model is shown as follows:

(16) $$\begin{array}{c} \underset{C}{\min}{ℒ}_{\text{Trans}C}=\underset{C}{\min}1-\overset{c}{\underset{i=1}{\sum }}\underset{c\in C}{\sum }\frac{\exp\left(-{\left\|C^{T}Y_{c}-C^{T}{\hat{Y}}_{ci}\right\|}_{2}^{2}\right)}{\sum_{l}\exp\left(-{\left\|C^{T}Y_{c}-C^{T}{\hat{Y}}_{ci}\right\|}_{2}^{2}\right)}+\theta_{3}^{{}^{\circ}},\\ \underset{C}{\text{min}}\underset{\left(Y_{c},{\hat{Y}}_{\mathrm{ci}}\right)\in ℳ}{\sum }{\left\|Y_{c}-{\hat{Y}}_{ci}\right\|}_{M}^{2},\\ \text{s.t}.\underset{\left(Y_{c},{\hat{Y}}_{c}\right)\in C}{\sum }{\left\|Y_{c}-{\hat{Y}}_{c}\right\|}_{M}^{2}\geq 1,\;M\geq 0. \end{array}$$

#### 3.5.3. Joint Loss Function

In the training process, to effectively supervise the feature loss caused by local convolution of the knowledge map and the partial filtering loss. When the divergence fusion crosses, the two tasks in the model are combined for training. This can improve the end-to-end training of the model. In summary, the joint loss function is written as

(17) $$\begin{array}{c} {ℒ}_{\text{Trans}C-GCN}={ℒ}_{Emb}+\gamma {ℒ}_{GCN}+\left(1-\gamma \right){ℒ}_{\text{Trans}C}+\theta^{{}^{\circ}}, \end{array}$$

where *γ* ∈ [0,1] is a hyperparameter that adjusts the ratio of balanced coding and partial crossover and *θ*°={*θ*_1_°, *θ*_2_°, *θ*_3_°} is the adjustment parameter.

## 4. Experiments

To further verify the effectiveness of TransC-GCN, we adopt the same experimental setting of Bordes et al. [24] in terms of entity prediction. In the evaluation index, the average ranking mean rank (MRR) and 10-hits rate (HITS@10) predicted by the entity are considered. According to the experience of Shimaoka et al. [25], we use the pretrained word vector as the initialization and optimize the parameters with the optimizer Adam [26]. We use TransC-GCN to generate the representation vector of the triple. To avoid overfitting, we add dropout to the neurons of GCN and randomly inactivate neurons of the vector iteration.

Furthermore, we compare our model with multiple baseline models under different parameter settings on the two tasks of entity type classification and entity attribute prediction. Moreover, we compare it with the baseline model [27], where ConvKB(https://github.com/daiquocnguyen/ConvKB) and ConnectE-E2T + TRT(https://github.com/Adam1679/ConnectE) programs were run.

### 4.1. Datasets

In order to be more pertinent and comparative, we refer to the datasets extracted from the text relationship [28] as our research object. The characteristics of the three datasets are shown in Table 1.

The visualization of the dataset intuitively shows that the number of entities and relationships and the degree of association have a greater impact on the local knowledge graph.  Figure 8 shows that in the three datasets, the entities and relationships of YAGO43kET are dense and rich. On the contrary, WN18 has sparse entities and lacks relationships.

### 4.2. Evaluation Index

In order to verify TransC-GCN, we refer to two typical evaluation methods [31]. Formally, mean reciprocal rank (MRR) is defined as

(18) $$\begin{array}{c} MRR=\frac{1}{\left|N\right|}\overset{n}{\underset{i=1}{\sum }}\frac{1}{{\text{Rank}}_{i}}, \end{array}$$

where *N* is the triplet number for the training dataset; *Rank*_*i*_ is the score averaged to the *i*th correct classification entity; and Hit rate is H_@K (*K* = 1/3/10), which means that in traversal training, the ability to obtain the correct triple entity prediction classification can be obtained once in *K* replacements.

### 4.3. Model Parameters

We conducted experiments on the training sets and the validation sets, as shown in Table 2.

We conducted cross explorations of different combinations in the setting of various parameters. According to the validation set effect of the corresponding dataset, the average ranking score will be the best.

### 4.4. Classification Prediction

Compared with tail entity and head entity prediction baseline models of the Bilinear, MLP and Trans series are shown in Table 3. WN18RR with dense entities and poor relationships and YAGO43kET with dense entities and rich relationships are selected. For relationship prediction verification, sparse entities and rich relationships of FB15kET are used.

#### 4.4.1. Entity Prediction

As shown in Figures 9 and 10, TransC-GCN is better than the compared entity prediction models in both recall and quality indicators. The aggregation and intersection of key paths on the local knowledge graph can effectively improve the efficiency and quality of node prediction. Prediction index results of the head entity and tail entity of the triple completion are close to each other, which shows that the aggregation of critical paths based on local graphs has strong applicability for node prediction.

#### 4.4.2. Relationship Prediction

Figure 11 shows that TransC-GCN also performs well in predicting the recall rate and quality of relationship evaluation. It not only considers the relationship path but also, more importantly, learns the characteristics of the knowledge graph through GCN, which can eliminate the random prediction of the model probability caused by the lack of triple entities or relationships to a certain extent. This provides richer necessary information for relationship path and entity prediction.

#### 4.4.3. Robustness

As shown in Figure 12, on the same dataset, two different training optimization methods of TransC-GCN_SGD and TransC-GCN_AdaGrad are compared. We can observe from Table 4 and Figure 13 that the number of entities and the number of relationships have a significant impact on the convolution and crossover of local knowledge graphs. In addition, the comparison result proves that the maximum pooling is indeed better than the average pooling in solving feature redundancy. In a graph with sparse entities and lack of relationships, there is a serious data sparse problem, which leads to the long-tail distribution of entities and relationships. However, we take advantage of the critical path in the local graph, and the structure of the global graph is used.

### 4.5. Case Study

We have shown that our TransC-GCN can handle large-scale knowledge graph and entity-relationship representation learning. In Figure 14, we provide an example of cross inference about local relationship paths. The core entity Savannah James is found through local cross learning. Two weak-strength relations (pay attention or like) are obtained by reasoning. We can find that Savannah James likes the 23 athletic undergarment bra of Zoe Saldana.

Because Savannah James like Zoe Saldana, she appreciated Avatar. Maybe she likes the bra of Athletic undergarment, which is of the brand Zoe Saldana. Of course, Savannah James must pay more attention to the player number of 23, so she may be want a signed 23 athletic undergarment bra of Zoe Saldana.

## 5. Conclusion and Future Work

In this paper, we propose a TransC-GCN method based on local convolution and global crossover for knowledge graph completion. ①This is the first time that local GCN and TransC are combined for knowledge graph representation learning. ②TransC-GCN can not only divide the huge knowledge graph into several local knowledge graphs and use convolutional neural network coding for more intelligent and subtle local knowledge graph feature learning with strong semantic relations but also realize the volume of adjacent nodes and relationship features. ③Pooling and filtering data noise provide a new and efficient method for node relationship prediction and classification. ④TransC-GCN considers the information value of nearby local knowledge graphs. We propose a parallel method of cross fusion of local knowledge graphs based on divergence, which combines local knowledge graphs and global knowledge graphs more flexibly in representation learning. In a number of challenging baseline model test comparisons. TransC-GCN has excellent performance in entity reasoning accuracy and generalization ability and is lightweight. However, there are deficiencies in entity diversity learning:

1. When the gradient adopts AdaGrad to start training, the square of the accumulated gradient is found, which causes the effective learning rate of GCN to decrease prematurely and excessively. After inactivating neurons with small gradients, ReLU is used as the activation function, resulting in loss of diversity.
2. Although experiments show that there is no significant difference between the maximum pooling and the average pooling in the results, there is still a loss of sparse entities in the test.
3. TransC-GCN is not efficient due to repeated calculations of neighbor nodes across subgraphs.

For future work, we will try to combine the pattern sequence ordering and the graph context to optimize TransC-GCN. Meanwhile, based on TransC-GCN, we intend to propose a new scene recommendation algorithm based on the combination of graph embedding and collaborative filtering.

## Figures and Tables

**Figure 1:** Node types and node predictions in the knowledge graph.

**Figure 2:** Local reasoning based on neighbor nodes and multihop reasoning in local graphs. (a) Mechanism 1. Infer potential nodes through neighbor nodes. (b) Mechanism 2. Through multihop key relationships in local knowledge graph.

**Figure 3:** Schematic diagram of using multiple local knowledge graphs for cross inference and completion of triples.

**Figure 4:** The local sampling and aggregation process of the graph.

**Figure 5:** End-to-end knowledge graph convolution cross embedding representation frame.

**Figure 6:** Predicting entities/relationships through multipart graph division and cross convolution.

**Figure 7:** Partial relationship diagram of the convolutional coding process.

**Figure 8:** Sparse visualization of dataset entities and relationships. (a) Dense entities and lack of relationships of YAGO43k/WN18RR. (b) Dense entities and rich relationships of YAGO43kET. (c) Sparse entities and lack of relationships of WN18. (d) Sparse entities and rich relationships of FB15kTRT/FB15kET.

**Figure 9:** Comparison of baseline models for tail entity prediction.

**Figure 10:** Comparison of baseline models for head entity prediction.

**Figure 11:** Comparison of relationship prediction of baseline models.

**Figure 12:** Robustness comparison of relationship prediction model on three datasets.

**Figure 13:** Comparison of baseline models of entity type prediction accuracy.

**Figure 14:** Entity node reasoning of user-commodity knowledge graph based on TransC-GCN.

**Algorithm 1:** Subgraph generation algorithm.

**Table 1:** Comparison of characteristics of different datasets.

Dataset	#Ent	#Rel	#Train	#Valid	#Test
FB15k [24]	14,951	1,345	483,142	50,000	59,071
WN18RR [29]	40,943	18	141,442	2,500	2,500
YAGO43k [30]	42,335	37	331,687	29,599	29,593
FB15kET	14,951	3,851	136,618	15,749	15,780
WN18R	40,501	10	110,341	2,100	2,100
YAGO43kET	41,723	45,182	375,853	42,739	42,750
FB15kTRT	3,851	1,345	2,015,338	—	—
YAGO43kTRT	45,128	37	1,727,707	—	—
WN18-R	6,501	5	90,341	—	—

**Table 2:** The optimal parameter configuration of the corresponding datasets.

Parameters	Datasets		
	YAGO43kET	WN18RR	FB15kET
*α*	0.1	0.1	0.1
*γ*	0.6	0.5	0.4
*q*	200	150	250
*ℓ*	100	100	125
Batch size	4096	4096	4096
Epochs	300	300	300

**Table 3:** Comparison of the overall effect of multiple baseline models on different datasets.

Dataset		YAGO43kET				WN18RR				FB15kET			
Metrics		MRR	H_@1	H_@3	H_@10	MRR	H_@1	H_@3	H_@10	MRR	H_@1	H_@3	H_@10
Methods	TransE	0.21	12.63	23.24	38.93	0.14	8.14	13.27	19.56	0.45	31.51	51.45	73.93
	TransE-ET	0.18	9.19	19.41	35.58	0.16	8.32	14.31	21.22	0.46	33.56	52.96	71.16
	TransR	0.19	10.23	19.97	36.75	0.16	8.44	17.92	26.71	0.47	34.63	53.67	72.02
	ETE	0.23	13.73	26.28	42.18	0.18	9.12	18.21	27.13	0.50	38.51	55.33	72.93
	PTransE	0.24	13.74	26.36	42.33	0.20	10.38	20.32	29.33	0.53	39.87	56.47	73.51
	ConnectE-(E2T+0)	0.25	13.66	26.38	44.60	0.21	11.71	23.31	30.74	0.57	45.82	62.60	80.01
	ConnectE-(E2T + TRT)	0.29	16.13	30.98	47.99	0.23	12.17	23.79	31.03	0.59	49.611	64.69	80.03
	TransC-GCN _AdaGrad	0.29 ± .32	17.12 ± .03	31.33 ± .21	48.72 ± .02	0.23 ± .21	13.76 ± .01	28.35 ± .13	33.07 ± .08	0.61 ± .03	49.47 ± .76	65.25 ± .44	81.02 ± .41
	TransC-GCN _SGD	0.29 ± .26	17.06 ± .17	30.95 ± .36	48.98 ± .00	0.24 ± .32	13.98 ± .36	29.18 ± .27	43.53 ± .03	0.61 ± .37	49.53 ± .40	65.39 ± .68	81.33 ± .32

**Table 4:** Comparison of baseline models of entity type prediction accuracy.

Dataset	YAGO43kET (%)	FB15kET (%)	WN18RR (%)
TransE	85.36	92.15	75.04
TransE-ET	90.76	93.23	77.13
PTransE	88.53	92.79	78.25
ETE	90.82	94.01	79.31
ConnectE-(E2T+0)	91.78	94.45	81.07
ConnectE-(E2T + TRT)	92.33	94.49	81.22
TransC-GCN_ AdaGrad	91.63	94.61♣	83.27
TransC-GCN_ SGD	92.75♣	94.58	84.55♣

## Data Availability

Some or all data, models, and codes generated or used during the study are available from the corresponding author upon request.
